The article "Nanocarbon Tracer and Areola Injection Site Are Superior in the Sentinel Lymph Node Biopsy Procedure for Breast Cancer" was retracted in 2023. Reasons: unreliable results or conclusions; lack of ethics approval or compliance; concerns about the data; concerns about the peer review.

# Nanocarbon Tracer and Areola Injection Site Are Superior in the Sentinel Lymph Node Biopsy Procedure for Breast Cancer

**DOI:** 10.1155/2022/4066179

**Published:** 2022-03-14

**Authors:** Bo Song, Binming Zhang, Aihu An, Yue Bai, Bo Gao

**Affiliations:** ^1^Department of Breast Surgery, Gansu Province Tumor Hospital, Lanzhou, 730050 Gansu, China; ^2^Department of Thoracic Surgery, Gansu Province Tumor Hospital, Lanzhou, 730050 Gansu, China

## Abstract

**Background:**

Axillary lymph node (ALN) staging is the most effective method to evaluate the condition of patients with breast cancer, their choice of treatment options, and prognosis. The sentinel lymph node (SLN) status assessment is the key to sentinel lymph node biopsy (SLNB) in patients with breast cancer. The choice of tracer and tracer injection sites affects SLNB.

**Objective:**

This study mainly analyzes the best tracer for SLNB and the best choice of tracer injection site.

**Methods:**

A total of 165 breast cancer patients who underwent SLNB were selected and injected with methylene blue or 99mTc-labeled sodium phytate or nanocarbon 20 min before biopsy. The number of SLNs detected by different tracers in different injection sites such as peritumoral tissue (PT) and subareolar area (SA) was counted, and the sensitivity, specificity, and positive/negative prediction rates were recorded and compared.

**Results:**

The detection success rate, average detection number of SLNs, and detection accuracy of the nanocarbon tracer were higher than the other two. The detection sensitivity, specificity, and positive and negative prediction rates of nanocarbon for SLNB were also higher than those of the other two tracers. When comparing the performance of tracers in different injection sites, it was found that the detection of three tracers injected in the SA was better than the injection in the PT.

**Conclusion:**

For women with early-stage breast cancer, nanocarbon can be used as the preferred tracer for SLNB to determine the status of the patient's ALNs, and the areola area can be used as the best injection site.

## 1. Introduction

Breast cancer endangers the lives and health of more than 20% of women worldwide and has the highest morbidity and mortality among women over 35 years of age [1, 2]. With the advances in early diagnostic technology, the prognosis of patients with breast cancer has improved significantly. However, breast cancer still inflicts more than 1 million new cases and causes over 400,000 deaths worldwide each year [3, 4]. Surgery is currently the mainstay of treatment for breast cancer, to remove tumor lesions located in the breast and axilla. Primary breast tumor treatment is based on radical mastectomy, whereas axillary treatment is based on axillary lymph node dissection (ALND) [5]. Lymph node metastasis is one of the main causes of death in patients with breast cancer. During ALND, axillary lymph nodes (ALNs) can be staged while removing potential metastatic lymph nodes, which is of great significance to improve the evaluation of the condition of patients, and better understand the treatment options and patient outcomes [6, 7]. Among patients with breast cancer who are detected at the early stages, only a small percentage develops ALN metastasis. ALND is not beneficial for patients without lymph node metastasis and may even cause adverse reactions such as lymphedema, sensory dysfunction, upper limb dysfunction, and lymphangiosarcoma [8, 9]. Therefore, doctors and scholars are exploring new methods to replace ALND in the determination of cancer metastasis in patients with breast cancer. With the same vision, this study hopes to contribute to the improvement of the survival rate of breast cancer patients.

The sentinel lymph node (SLN) is the first lymph node that the primary tumor must pass through for metastasis and is an effective barrier against tumor cell metastasis [10]. Since the application of SLN biopsy (SLNB) in breast cancer surgery in the 1990s, ALND in patients with negative ALNs had been avoided, contributing to improved quality of life of patients [11, 12]. With the further development of tracing technology in recent years, SLNB can accurately locate a patient's SLN and predict the ALN status. Therefore, SLNB has replaced ALND as the primary method to determine lymphatic metastasis in patients with early-stage breast cancer. The tracer and injection site are of great importance when it comes to lymphatic dissection for patients with breast cancer, as different tracers and injection sites directly affect the diagnosis. Although several studies have confirmed the feasibility and reliability of SLNB in the diagnosis of ALN metastasis in patients with early-stage breast cancer, the choice of tracer and injection site for SLNB remains controversial. Currently, the commonly used SLNB tracers include biological dyes, radionuclides, and nanocarbon, each of which has its advantages and disadvantages. Among them, biological dye tracers have the lowest sensitivity. While the radionuclides have the highest sensitivity, they require a laparoscope with fluorescence function to work. Nanocarbon, with the smallest diameter, can quickly enter the lymphatic vessels, enhancing the contrast between the lymphatic vessels and the surrounding tissues. However, there remains a dearth of knowledge regarding the effectiveness of nanocarbon in SLNB [13–15].

Previous studies have shown that injecting tracers around breast cancer tumor tissues can accurately reflect the true conditions of tumor tissue, which intuitively makes peritumoral tissue (PT) the first choice for early SLNB tracer injection. However, in long-term clinical practice, it has been found that tracer injection into the PT requires the coordination of ultrasound or other imaging instruments, which increases the cost by requiring an imaging operator and the time required to complete the procedure. In addition, due to the presence of tumor tissue in the tissue surrounding the tumor, the visualization effect of the tracer on PT will be affected by the extent and depth of infiltration. Therefore, to more accurately locate and identify the status of SLNs in patients with breast cancer, it is necessary to find a new tracer injection site for SLNB. In recent years, scholars have proposed that the areola area is rich in lymphatic vascular plexus, which has a greater advantage for tracer visualization in SLNB [16]. Scholars such as Wärnberg pointed out that choosing the subareolar area (SA) as the tracer injection site can increase the detection rate, providing a new SLNB tracer injection site [17]. There are still controversies over the various choices of tracers and their injection sites, as well as whether the detection combing tracers and injection sites can achieve the best results. Therefore, this study compares the effects of different tracers and different injection sites on the detection accuracy of SLNB in breast cancer, hoping to resolve the controversy over the selection of SLNB tracers and injection sites for breast cancer.

## 2. Materials and Methods

### 2.1. Research Subjects

This study has been approved by the Ethics Committee of Gansu Province Tumor Hospital. One hundred and sixty-five patients who underwent SLNB for breast cancer in Gansu Province Tumor Hospital from January 2019 to December 2020 were selected as research participants. Inclusion criteria are as follows: (1) diagnosis of unilateral breast invasive carcinoma by puncture pathological examination, (2) TNM staging: CTis-2N0M0, (3) no serious medical disease, (4) age < 70 years, and (5) the primary tumor is a single lesion. Exclusion criteria are as follows: (1) male; (2) use of adjuvant therapy such as radiotherapy, chemotherapy, or endocrine therapy before enrollment; (3) women who are pregnant or breastfeeding; and (4) allergies to the tracers used in this study. All participants were informed of the purpose of this study and provided informed consent.

### 2.2. Grouping

According to the type and location of the tracer injected, patients were divided into methylene blue+peritumoral tissue (MB+PT, *n* = 30), MB+subareolar area (MB+SA, *n* = 28), 99mTc-labeled sodium phytate and stannous chloride+PT (99mTc-PHY+PT, *n* = 29), 99mTc-PHY+SA (*n* = 26), nanocarbon+PT (CN+PT, *n* = 26), and CN+SA (*n* = 26) groups. The general information of patients was found to have no statically significant effect on the results and was therefore not included in the study, as shown in Table 1.

### 2.3. Intervention Methods

The intervention methods were as follows: In the MB+PT group, methylene blue was injected into the PT of the patient 20 minutes before the biopsy, with a total injection dose of 2 mL. The injection time and location of the MB+SA group were the same as those in the MB+PT group, but the total injection dose was 1.5 mL. The 99mTc-PHY+PT group received 0.4 mL per point in the tissue 12 hours before the biopsy. The injection time of the 99mTc-PHY+SA group was the same as that of the 99mTc-PHY+PT group, but the injection dose was changed to 0.2 mL in the high-risk affected areola area. The CN+PT group was injected with a nanocarbon suspension into the tissue around the affected tumor 12 hours before the biopsy, and the total injection dose was 2 mL. The CN+SA group had the same injection time and site as the CN+PT group, and the total injection dose was changed to 1 mL. After injection, each group was examined by a gamma-ray detector to detect the effect of SLN staining. Ten minutes after the completion of the injection, a 3 cm long dermatoglyphic incision was made in the second fold of the axillary skin on the injection side and the SLNB was performed. Pathological analysis of SLNs that were successfully stained during surgery was performed, based on which surgery was performed when necessary. Patients who were not successfully stained were treated with modified radical mastectomy for breast cancer.

### 2.4. Comparison of Detection Conditions

The number of SLNs detected by different tracers at different injection sites was counted; pathological examination results were used as the gold standard to analyze and compare the detection performance of different tracers. The detection sensitivity was calculated as the number of true positives measured by the target method divided by the number of true positives measured by the gold standard. The specificity was calculated as the number of true negatives measured by the target method divided by the number of true negatives measured by the gold standard. The accuracy rate was the sum of the number of true positives and true negatives measured by the target method divided by the sum of the number of true positives and true negatives measured by the gold standard. The positive prediction rate was the number of true positives measured by the target method divided by the number of positives measured by this method. The negative prediction rate was the number of true negatives measured by the target method divided by the number of negatives measured by this method.

### 2.5. Statistical Analysis

In this study, SPSS 25.0 (EASYBIO Technology Co., Ltd., Beijing, China) and GraphPad Prism 8.2 (Shanghai Universal Biotech Co., Ltd., Shanghai, China) were used for data analysis and image rendering, respectively. Quantitative data is expressed in the form of mean ± standard deviation; intergroup comparisons, multigroup comparisons, and pairwise comparisons between multiple groups were performed by *t*-test, analysis of variance, and SNA-*Q* test, respectively. Qualitative data is represented by *n* (%) and analyzed using the chi-square test. When the theoretical frequency was between 1 and 4, the corrected chi-square was used. Rank data was tested by a rank-sum test. Differences with *P* < 0.05 were considered statistically significant.

## 3. Results and Discussion

### 3.1. SLN Detection Success Rate and Average Detection Number of Different Tracers

Nanocarbon had the highest detection rate of SLNs, followed by 99mTc-PHY, and MB had the lowest when comparing the detection success rate of the three tracers with the average detection rate. Although statistical analysis showed no significant difference (*P* > 0.05), this may be due to the small sample sizes of this study. Further, the average number of SLNs detected by the different tracers was compared, and significant differences were found among the three tracers (*P* < 0.05). Among them, the average number of SLNs detected by nanocarbon was the highest (the specific data are shown in Table 2 and Figure 1).

### 3.2. Detection Values of MB Injected in Different Parts

To compare the effects of different injection sites on the detection of SLNs by SLNB, we compared the detection performance of the three tracers after injected them into the PT and the SA. First, the detection of MB in the PT and the SA were compared, as shown in Table 3. After analysis, it was found that the detection specificity, accuracy, and positive prediction rate in the SA was higher than those in the PT, but with no statistical significance (*P* > 0.05; Table 4 and Figure 2).

### 3.3. Detection Values of 99mTc-PHY Injected in Different Parts

The detection of 99mTc-PHY injected in the PT and the SA were compared (Table 5). The analysis showed that the specificity, accuracy, and positive and negative prediction rates of the detection sensitivity injected in the SA were higher than those in the PT, but the differences were not statistically significant (*P* > 0.05; Table 6 and Figure 3).

### 3.4. Detection Values of Nanocarbon Injected in Different Parts

The detection of nanocarbon (the electron micrograph of nanocarbon is shown in Figure 4(a)) injection in the PT and the SA were compared (Table 7). After analysis, it was found that the detection sensitivity, specificity accuracy rate, and positive and negative prediction rates of injection in the SA were higher than those in the PT, but the differences were not statistically significant (*P* > 0.05; Table 8 and Figure 4(b)).

### 3.5. Detection Values of Different Tracers for SLNs by SLNB

The specific situation of SLNs detected by SLNB with different tracers was compared along with the pathological examination results (Table 9). After comparison and analysis, we found that the three tracers had great differences in the detection accuracy of SLNs in SLNB (*P* < 0.05), among which nanocarbon had the highest accuracy (*P* < 0.05). In addition to the detection accuracy rate, the sensitivity, specificity, and positive and negative prediction rates of nanocarbon for SLN detection in SLNB were also higher than those of MB and 99mTc-PHY, but without statistical significance (*P* > 0.05; Table 10 and Figure 5).

### 3.6. Discussion

Breast cancer mainly occurs in women with a high recurrence rate, posing a great threat to the life safety of patients. The main route of breast cancer metastasis is through lymph nodes. Most of the lymph nodes in the breast drain to the axilla, a small amount into the parasternal lymph nodes, and some into the supraclavicular lymph nodes [18, 19]. Since most breast lymph nodes metastasize to the axilla, ALN metastasis is an important indicator for evaluating the prognosis of patients with breast cancer. SLNB uses a tracer to locate the patient's SLNs, instructing clinicians to perform surgery. However, some studies have shown that different tracers and injection sites significantly affect the detection of SLNs by SLNB. Although studies have compared the effects of different tracers or injection sites for SLNB, there is currently no research to investigate the combined use of tracers and injection sites [20, 21]. Therefore, this study compares the effects of different tracers injected at different sites on the detection of SLNs, providing a reference for improving the detection success rate and accuracy of SLNB.

In this study, we compared the detection success rate and the average number of SLNs detected by SLNB using MB, 99mTc-PHY, and nanocarbon. The results showed that the detection success rate and the average number of SLNs detected by nanocarbon were higher than those of the other two. The detection values of the three tracers were further compared to reveal that the detection accuracy, sensitivity, specificity, and positive and negative prediction rates of nanocarbon for SLNs were all higher than the other two. And compared with methylene blue, the sensitivity of 99mTc-PHY was higher in the detection of SLNs. 99mTc-PHY is a radionuclide-labeled carrier, and those treated with it and handling it will be exposed to ionizing radiation. While studies have shown that the radionuclide dose and radiation intensity used in SLNB will not cause fatal harm to patients and doctors, the less radiation patient healthcare workers must be exposed to, the better. How radionuclide-labeled tracer affects the health of such personnel remains to be explored [22]. However, it is recognized that ionizing radiation can greatly interfere with the proliferation of animal cells [23]. Therefore, we believe that nanocarbon is a better alternative for the detection of SLNs in SLNB because it yields good detection results and is safer.

In the early stages of breast cancer, tumor tissue is often chosen as the tracer injection site for SLNB. However, in clinical practice, it is difficult for inexperienced injectors to accurately inject the tracer into the PT during surgery. In addition, for patients with inaccessible lesions, the injection of tracer into the PT needs to be completed with the assistance of an imaging personnel. Therefore, we believe that tracer injection into the PT requires knowledgeable medical staff, which complicates the biopsy procedure [24–35]. When comparing different injection sites in this study, it was found that the detection performance of the three tracers, MB, 99mTc-PHY, and nanocarbon, injected in the SA was better than that injected in the PT. Mehrabibahar et al. also proposed that the injection of tracers around the areola area could effectively locate the lymph nodes [36]. Therefore, we believe that when performing SLNB, nanocarbon can be used as a preferred tracer, using the areola as the best injection site. The role of nanocarbon tracers in predicting lymph node metastasis in cancer has also been previously demonstrated. For example, Wang et al. [37] reported that nanocarbon tracers can help surgeons accurately remove SLNs during laparoscopic colorectal cancer surgery and improve patient outcomes. In addition, Wang et al. [38] pointed out that nanocarbon can also be used as a suspension to help improve the detection rate of lymph nodes in early oral squamous cell carcinoma, which has a certain guiding role in the treatment of the disease.

The novelty of this study is as follows: (1) by comparing the detection success rate and average detection number of SLNs with methylene blue, 99mTc-labeled sodium phytate, and nanocarbon, it is confirmed that nanocarbon is the most advantageous among the three tracers; (2) by comparing the performance of the three tracers in different injection sites, it is identified that the tracers are more effective in the SA than in the PT.

However, this study was affected by the low sample size, which resulted in no statistically significant differences in many of the indicators. Second, no adverse effects were observed in this study, which may also require studies with larger samples to make a correct assessment. Third, the analysis of the combined diagnosis of breast cancer with two tracers could provide new insights into the tracer management of breast cancer. We will conduct in-depth research from the above aspects in future studies to verify the experimental results.

## 4. Conclusion

In summary, this study compared the effects of three tracers on the detection of SLNs in SLNB and found that the detection success rate and average number of SLNs detected by nanocarbon were the highest. In addition, the detection accuracy of the three tracers differs greatly, with that of nanocarbon being the most accurate. The detection sensitivity, specificity, and positive and negative prediction rates of nanocarbon in SLNB for SLNs were also higher than those of the other two tracers. The effects of different injection sites on the detection of SLNs were also investigated, and it was found that the detection values of the three tracers injected in the SA were higher than those in the PT. Therefore, when performing SLNB, nanocarbon should be used as the preferred tracer and the SA as the best tracer injection site.

## Figures and Tables

**Figure 1:** Effects of different tracers on SLNB. (a) The detection success rate of different tracers. (b) Average number of SLNs detected by different tracers. ^∗^*P* < 0.05.

**Figure 2:** Comparison of the detection value of the methylene blue injection in different areas.

**Figure 3:** Comparison of the value of the 99mTc-PHY injection in different areas.

**Figure 4:** Electron micrograph of nanocarbon tracer and its diagnostic value for breast cancer. (a) The electron micrograph of nanocarbon. (b) The diagnostic value of the nanocarbon injection in different areas.

**Figure 5:** Comparison of the value of different tracers in the detection of SLNs by SLNB.

**Table 1:** General data distribution and comparison of patients in each group.

Groups	Age (years)	Tumor location		Quadrant			
		Left	Right	Upper	Outer	Inner upper	Inner outer
MB+PT	47.62 ± 9.72	19 (63.33)	11 (36.67)	19 (63.33)	4 (13.33)	5 (16.67)	2 (6.67)
MB+SA	49.18 ± 10.22	13 (46.43)	15 (53.57)	18 (64.29)	2 (7.14)	4 (14.29)	4 (14.29)
99mTc-PHY+PT	48.63 ± 10.27	16 (55.17)	13 (44.83)	20 (68.97)	2 (6.90)	4 (13.79)	3 (10.34)
99mTc-PHY+SA	49.64 ± 9.82	16 (61.54)	10 (38.46)	17 (65.38)	3 (11.54)	2 (7.69)	4 (15.38)
CN+PT	47.91 ± 10.28	17 (65.38)	9 (34.62)	18 (69.23)	2 (7.69)	1 (3.85)	5 (19.23)
CN+SA	46.86 ± 10.96	14 (53.85)	12 (46.15)	16 (61.54)	4 (15.38)	2 (7.69)	4 (15.38)
F/X^2^	0.275	2.864		7.089			
*P*	0.926	0.721		0.955			

**Table 2:** Comparison of the SLN detection success rate and average detection number of different tracers.

Tracer material	Detection success rate	Average number of detected
Methylene blue	86.21 (50/58)	3.10 ± 0.71
99mTc-PHY	90.91 (50/55)	3.30 ± 0.76
Nanocarbon	96.15 (50/52)	3.46 ± 0.68^∗^
*F*	3.282	3.160
*P*	0.194	0.045

Note. ∗ represents compared with methylene blue groups, *P* < 0.05.

**Table 3:** Effects of methylene blue injection at different sites on the detection of SLNs.

Injection site	Methylene blue detection	Histopathologic test		Total
		Positive	Negative	
PT	Positive	7	6	13
	Negative	4	8	12
	Total	11	14	25
SA	Positive	7	4	11
	Negative	4	10	14
	Total	11	14	25

**Table 4:** Comparison of the value of methylene blue injection in different parts.

Tracer material	Sensitivity	Specificity	Accuracy rate	Positive prediction rate	Negative prediction rate
PT	63.64 (7/11)	57.14 (8/14)	60.00 (15/25)	53.85 (7/13)	66.67 (8/12)
SA	63.64 (7/11)	71.43 (10/14)	68.00 (17/25)	63.64 (7/11)	71.43 (10/14)
*χ* ^2^	0.000	0.622	0.347	0.235	0.069
*P*	1.000	0.430	0.556	0.628	0.793

**Table 5:** Effects of the 99mTc-PHY injection at different sites on the detection of SLNs.

Injection site	99mTc-PHY detection	Histopathologic test		Total
		Positive	Negative	
PT	Positive	8	4	12
	Negative	3	10	13
	Total	11	14	25
SA	Positive	9	3	12
	Negative	2	11	13
	Total	11	14	25

**Table 6:** Comparison of the value of the 99mTc-PHY injection in different parts.

Tracer material	Sensitivity	Specificity	Accuracy rate	Positive prediction rate	Negative prediction rate
PT	72.73 (8/11)	71.43 (10/14)	72.00 (18/25)	66.67 (8/12)	76.92 (10/13)
SA	81.82 (9/11)	78.57 (11/14)	80.00 (20/25)	75.00 (9/12)	84.62 (11/13)
*χ* ^2^	0.259	0.190	0.095	0.202	0.026
*P*	0.611	0.663	0.758	0.653	0.871

**Table 7:** Effects of the nanocarbon injection at different sites on the detection of SLNs.

Injection site	Nanocarbon detection	Histopathologic test		Total
		Positive	Negative	
PT	Positive	9	2	11
	Negative	2	12	14
	Total	11	14	25
SA	Positive	10	2	12
	Negative	1	12	13
	Total	11	14	25

**Table 8:** Comparison of the value of the nanocarbon injection in different parts.

Tracer material	Sensitivity	Specificity	Accuracy rate	Positive prediction rate	Negative prediction rate
PT	81.82 (9/11)	85.71 (12/14)	84.00 (21/25)	81.82 (9/11)	85.71 (12/14)
SA	90.91 (10/11)	85.71 (12/14)	88.00 (22/25)	83.33 (10/12)	92.31 (12/13)
*χ* ^2^	0.386	0.000	0.166	0.253	0.297
*P*	0.534	1.000	0.684	0.615	0.586

**Table 9:** Detection results of SLNs by SLNB with different tracers.

Tracer material		Histopathologic test		Total
		Positive	Negative	
Methylene blue detection	Positive	14	10	24
	Negative	8	18	26
	Total	22	28	50
99mTc-PHY detection	Positive	17	7	24
	Negative	5	21	26
	Total	22	28	50
Nanocarbon detection	Positive	19	3	22
	Negative	3	25	28
	Total	22	28	50

**Table 10:** Comparison of the value of different tracers in the detection of SLN by SLNB.

Tracer material	Sensitivity	Specificity	Accuracy rate	Positive prediction rate	Negative prediction rate
Methylene blue	63.64 (14/22)	64.29 (18/28)	64.00 (32/50)	58.33 (14/24)	69.23 (18/26)
99mTc-PHY	77.27 (17/22)	75.00 (21/28)	76.00 (38/50)	70.83 (17/24)	80.77 (21/26)
Nanocarbon	86.36 (19/22)	89.29 (25/28)^∗^	88.00 (44/50)^∗^	86.36 (19/22)^∗^	89.29 (25/28)
*χ* ^2^	3.135	4.856	7.895	4.425	2.454
*P*	0.209	0.088	0.019	0.109	0.293

Note. ^∗^Compared with methylene blue group, *P* < 0.05.

## Data Availability

The simulation experiment data used to support the findings of this study are available from the corresponding author upon request.
